The article "Patients with Griscelli syndrome and normal pigmentation identify RAB27A mutations that selectively disrupt MUNC13-4 binding" was published in 2015. Journal: J Allergy Clin Immunol.

# Patients with Griscelli syndrome and normal pigmentation identify *RAB27A* mutations that selectively disrupt MUNC13-4 binding

**DOI:** 10.1016/j.jaci.2014.08.039

**Published:** 2015-05

**Authors:** Valentina Cetica, Yvonne Hackmann, Samantha Grieve, Elena Sieni, Benedetta Ciambotti, Maria Luisa Coniglio, Daniela Pende, Kimberly Gilmour, Paolo Romagnoli, Gillian M. Griffiths, Maurizio Aricò

**Affiliations:** a Pediatric Hematology Oncology, Azienda Ospedaliero–Universitaria Meyer Children's Hospital, Florence, Italy; b Cambridge Institute for Medical Research, University of Cambridge Biomedical Campus, Addenbrooke's Hospital, Cambridge, United Kingdom; c Istituto di Ricovero e Cura a Carattere Scientifico Azienda Ospedaliera Universitaria San Martino–Istituto Nazionale per la Ricerca sul Cancro, Genoa, Italy; d Immunology, Great Ormond Street Hospital, London, United Kingdom; e Department of Experimental and Clinical Medicine, University of Florence, Florence, Italy; f Pediatric Oncology Network, Istituto Toscano Tumori (I.T.T.), Florence, Italy

**Keywords:** Hemophagocytic lymphohistiocytosis, familial hemophagocytic lymphohistiocytosis, Griscelli syndrome type 2, melanophilin, cytotoxic T lymphocyte, natural killer cells, CTL, Cytotoxic T lymphocyte, FHL, Familial Hemophagocytic lymphohistiocytosis, GFP, Green fluorescent protein, GRA, Granule release assay, GS2, Griscelli syndrome type 2, GTP, Guanosine triphosphate, HLH, Hemophagocytic lymphohistiocytosis, Mlph, melanophilin, NK, Natural killer, OMIM, Online Mendelian Inheritance in Man, Slp2a, Synaptotagmin-like protein 2a

## Abstract

**Background:**

Familial hemophagocytic lymphohistiocytosis (FHL) is a rare and often fatal disorder characterized by defective cellular cytotoxicity and hyperinflammation, and the only cure known to date is hematopoietic stem cell transplantation. Mutations in *RAB27A*, *LYST*, and *AP3B1* give rise to FHL associated with oculocutaneous albinism, and patients with FHL are usually only screened for mutations in these genes when albinism is observed. A number of patients with FHL and normal pigmentation remain without a genetic diagnosis.

**Objective:**

We asked whether patients with FHL with immunodeficiency but with normal pigmentation might sometimes have mutations that affected cellular cytotoxicity without affecting pigmentation.

**Methods:**

We carried out mutation analysis of *RAB27A*, *LYST*, and *AP3B1* in patients with FHL with pigment dilution, as well as a cohort with no clinical evidence of pigment dilution but no mutations in the other known FHL-related genes (*PRF1*, *STXBP2*, and *UNC13D*).

**Results:**

We identify patients with Griscelli syndrome type 2 with biallelic mutations in *RAB27A* in the absence of albinism. All 6 patients carried mutations at amino acids R141, Y159, or S163 of Rab27a that disrupt the interaction of Rab27a with Munc13-4, without impairing the interaction between melanophilin and Rab27a.

**Conclusion:**

These studies highlight the need for *RAB27A* sequencing in patients with FHL with normal pigmentation and identify a critical binding site for Munc13-4 on Rab27a, revealing the molecular basis of this interaction.

Familial hemophagocytic lymphohistiocytosis (FHL; Online Mendelian Inheritance in Man [OMIM] 267700) is a genetically heterogeneous disorder characterized by a hyperinflammatory syndrome with fever, hepatosplenomegaly, cytopenia, and sometimes central nervous system involvement. Bone marrow aspiration is usually performed early during the diagnostic work-up, enabling the identification of hemophagocytosis by activated macrophages. In most cases the natural course of FHL is rapidly fatal within a few weeks unless appropriate treatment, including corticosteroids, cyclosporine, etoposide, and anti-thymocyte globulin, results in transient disease control.^1^ To date, only patients undergoing hematopoietic stem cell transplantation have been cured.^1-6^ FHL is associated with hyperactivation of the immune system, which is thought to result from the failure of activated cytotoxic T lymphocytes (CTLs) and natural killer (NK) cells to clear virally infected cells and terminate the immune response. The failure to clear virally infected cells is thought to lead to the activation and uncontrolled expansion of polyclonal CD8^+^ T cells and give rise to macrophage activation, with infiltration of tissues and organs, excessive release of inflammatory cytokines, and resultant tissue damage.^7,8^

Diagnosing FHL has remained a challenge for many years. Initially, the diagnostic criteria established by the Histiocyte Society were key and included a collection of both clinical and biochemical features. These diagnostic criteria have been updated to introduce hyperferritinemia, defective NK cell activity, and soluble CD25 levels.^9^ A better understanding of the pathogenic mechanisms of FHL has provided a rationale for developing novel, sensitive, and specific diagnostic tools based on flow cytometric analysis of peripheral blood cells, including defective expression of intracellular perforin and defective degranulation.^10,11^ However, the gold standard for diagnosing FHL remains mutational analysis of FHL-related genes. This is therapeutically vital in deciding whether patients should undergo hematopoietic stem cell transplantation^12,13^ and whether prenatal diagnosis is appropriate within families.

Since 1999, several genes have been associated with FHL: *PRF1* (OMIM *170280), *UNC13-D* (OMIM *608897), *STX11* (OMIM *605014), and *STXBP2* (OMIM *601717), all encoding proteins that play a key role in lymphocyte-mediated cytotoxicity.^14-17^ In addition, biallelic mutations in *RAB27A* (OMIM *603868)^18^ give rise to a form of FHL known as Griscelli syndrome type 2 (GS2). CTLs and NK cells from these patients show defective degranulation and target cell killing; in addition, these patients show partial oculocutaneous albinism with a silver-gray sheen of hair and large pigment aggregates of melanosomes within melanocytes in hair shafts. This combined phenotype arises as a result of Rab27a's ability to control both melanosome secretion from melanocytes and cytolytic granule secretion from CTLs.^19-22^ In melanocytes Rab27a mediates secretion by binding to the synaptotagmin-like protein melanophilin (Mlph), as well as the plus-end directed motor protein myosin Va, which delivers melanosomes to cortical actin for secretion.^22-25^ In CTLs Rab27a controls secretion of cytolytic granules by binding the priming factor Munc13-4,^15,26^ and mutations in either Munc13-4 or Rab27a prevent secretion of granules once they have reached the immunologic synapse formed between a CTL and a target cell. Interestingly, mutations in Munc13-4 do not affect melanocyte function, and mutations in Mlph do not give rise to FHL.^27,28^ In this way Rab27a controls secretion in 2 different cell types by interacting with different effector proteins.

Little is known about the precise sites of interaction between Rab27a and Munc13-4. Earlier work mapped the Rab27a-binding site on Munc13-4 to a motif spanning residues 280 to 285.^29^ However, this study did not pinpoint the key amino acids of Rab27a that facilitate the interaction with Munc13-4 or whether the same binding site mediates Rab27a interaction with Mlph. Because Munc13-4 interacts with Rab27a in the guanosine triphosphate (GTP)–bound state^30^ and the W73G mutation disrupts binding to Munc13-4 and Mlph, this suggests that changes around the GTP-binding site probably facilitate both interactions.

In this article we examine the link between FHL and pigmentation defects in 21 patients and identify novel mutations in *RAB27A*, *LYST*, *AP3B1*, and, surprisingly, *PRF1* in 1 patient. We have also discovered a newly defined subpopulation of patients with GS2 with mutations in *RAB27A* despite normal pigmentation. We show that the *RAB27A* mutations in these patients disrupt interaction with Munc13-4 but do not affect binding to Mlph. These mutations identify key amino acids required for interaction with Munc13-4 and reveal discrete binding sites for Munc13-4 and Mlph on Rab27a.

## Methods

### Patient cohort

In 1989, a registry for hemophagocytic lymphohistiocytosis (HLH) was established,^1^ with the aim of centralizing patient information and immunologic and genetic studies for diagnosis. HLH was defined by the diagnostic criteria established by the Histiocyte Society.^9^

Of 901 patients referred between 1989 and 2013, 795 (88%) were given a diagnosis of HLH. Of these, 592 underwent mutation analysis, which in 240 (40%) cases provided identification of a genetic diagnosis of FHL-related condition. Within this cohort, we selected all cases in which pigment dilution, identified by clinicians on the basis of hair color, was reported as part of the clinical picture. In addition, we retrospectively reviewed all patients in whom the final diagnosis was FHL but in whom a genetic marker could not be attributed. In such cases we decided to sequence the pigment dilution–related genes. Informed consent was obtained in all cases by the parents or legal guardian. The study was approved by the A.O.U. Meyer Institutional Review Board.

### Perforin expression and degranulation assays

PBMCs from patients with FHL and healthy donors were isolated by using Ficoll gradient centrifugation. Perforin expression in NK cells (CD3^−^CD56^+^ cells of PBLs) was detected by means of intracellular staining (after fixation and permeabilization) with the BD PharMingen (San Jose, Calif) reagent set and cytofluorimetric analysis, as previously reported.^31^

Resting and activated NK cells were also tested by using the granule release assay (GRA), quantifying cell-surface CD107a expression on coculture with K562, as previously described.^11,32,33^ Briefly, anti-CD107a–phycoerythrin mAb was added during the coculture for 3 hours at 37°C in 5% CO_2_. Thereafter, the cells were stained with anti-CD56–allophycocyanin and anti-CD3–peridinin-chlorophyll-protein complex mAb and analyzed by using flow cytometry (FACSCalibur, Becton Dickinson). All reagents were from BD Biosciences. Surface expression of CD107a was assessed in CD3^−^CD56^+^ cells (NK cells). Results were evaluated as ΔCD107a (ie, Percentage of CD107a^+^ cells of stimulated − Percentage CD107a^+^ cells of unstimulated sample) and defined as defective when lower than the 10th percentile of values in healthy control subjects.

### Cell culture

HEK 293 and P815 target cells were maintained in RPMI or Dulbecco modified Eagle medium, respectively (Gibco, Life Technologies, Grand Island, NY), supplemented with 10% FBS. Primary human CD8^+^ T cells were negatively selected from PHA blasts by using the Dynabeads Untouched Human CD8^+^ kit (Life Technologies), according to the manufacturer's instructions, and stimulated with irradiated (3000 rads) PBMCs and 1 μg/mL PHA (Oxoid, Hampshire, United Kingdom). Cells were grown in RPMI supplemented with 5% human serum, 100 U/mL recombinant IL-2, 1 mmol/L sodium pyruvate, 2 mmol/L l-glutamine, 0.075% sodium carbonate, and 50 μmol/L 2-mercaptoethanol to obtain CTLs. Polyclonal NK cell populations were also obtained after NK cell purification (RosetteSep Method; STEMCELL Technologies, Vancouver, British Columbia, Canada) and cultured, as previously described.^11^

### Cytotoxicity assays

CTLs and P815 target cells were resuspended in RPMI (without phenol red, Gibco), 2% FBS, and 0.5 μg/mL anti-CD3 antibody (clone UCHT1, BD Biosciences); plated at different effector/target ratios as shown; and incubated at 37°C for 4 hours. The CytoTox 96 kit (Promega, Madison, Wis) was used to assess target cell lysis per the manufacturer's instructions. Activated purified NK cells were tested for cytolytic activity against the 221 B-EBV target cell line in a standard ^51^Cr-release assay.^11^

### Biochemical studies

HEK 293 cells were lipofected (Lipofectamine 2000, Life Technologies) with full-length human Rab27a–green fluorescent protein (GFP) locked in its GTP-bound form by mutation Q78L with and without additional mutations A76V, Y159C, S163R, or p.R141_V142delinsI and either Munc13-4–GFP or Mlph-GFP.

Lipofected HEK 293 cells were lysed with PBS plus 1% Triton X-100, 4-(2-aminoethyl) benzenesulfonyl fluoride hydrochloride (AEBSF), 1 mmol/L CaCl_2_, and 1 mmol/L MgCl_2_. Lysates were precleared with 100 μL of Protein G Bead slurry (GE Healthcare, Fairfield, Conn) with rotating at 4°C for 30 minutes and then split into 3 samples: no antibody, rabbit anti-Rab27a (produced in rabbits immunized with human Rab27a-GST and screened against lysates from healthy donor and Rab27A-deficient human and mouse cell lines), and either goat anti–Munc13-4 (Everest Biotechnology, Upper Heyford, United Kingdom) or rabbit anti-Mlph (Abcam, Cambridge, United Kingdom). Lysates and antibodies were incubated for 2 hours with rotating at 4°C, followed by addition of Protein G beads and incubation for 1 hour. Beads were washed 4 times with lysis buffer, resuspended with sample buffer, and boiled at 95°C for 5 minutes, and the eluate was then transferred to a fresh tube.

Samples were separated on a 10% acrylamide gel and transferred onto nitrocellulose. Membranes were blocked in PBS with 0.2% Tween 20 and 5% dried skim milk powder and incubated with primary antibodies (as used in IP plus mouse anti-Rab27a [Abnova, Taipei City, Taiwan] or rabbit anti-Mlph [Proteintech, Chicago, Ill]). Membranes were washed 3 times for 10 minutes with PBS plus 0.2% Tween 20 and incubated in secondary antibodies conjugated to horseradish peroxidase (HRP; anti-goat HRP, anti-mouse HRP, and anti-rabbit light chain–specific HRP; all from Jackson ImmunoResearch, West Grove, Pa), washed again as before with an additional 10-minute wash with PBS alone, and then developed with UptiLight (Cheshire Sciences, Chester, United Kingdom) and exposed on x-ray film (Kodak, Rochester, NY).

### Pigmentation analysis

Hair samples were cleared in xylene, mounted with synthetic resin (Eukitt; Fluka, Sigma-Aldrich, St Louis, Mo), and observed under a Leitz (Wetzlar, Germany) light microscope equipped with a ProgRes C10plus camera and dedicated software (Jenoptik, Jena, Germany).

### Mutation analysis

Genomic DNA was isolated from peripheral blood samples by using the BioRobot EZ1Workstation (Qiagen, Hilden, Germany). *RAB27A*, *LYST*, *AP3B1*, and *PRF1* genes were analyzed by means of direct sequencing. The coding exons and exon-intron boundaries were amplified and directly sequenced in both directions with the BigDye Terminator Cycle Sequencing Ready Reaction Kit (Applied Biosystems, Foster City, Calif). Sequences obtained with an ABI Prism 3130XL Sequence Detection System (Applied Biosystems) were analyzed and compared with the reported gene structure by using the dedicated software SeqScape (Applied Biosystems). All mutations were confirmed in the parents.

### *In silico* analysis

All variants of the sequence were searched in dbSNP (http://www.ncbi.nlm.nih.gov/snp/). For variants not reported, we used 3 bioinformatics tools to predict whether an amino acid substitution could be benign or deleterious: SIFT (Sorting Intolerant From Tolerant; http://sift.jcvi.org/), PolyPhen (Polymorphism Phenotyping; http://genetics.bwh.harvard.edu/pph/), and Pmut (http://mmb.pcb.ub.es/Pmut).^34^

## Results

### Patients with FHL with partial albinism with assigned genetic markers

A total of 21 children from 20 families were reported to have HLH and some degree of pigment dilution. They accounted for 2.5% of the total cases of HLH enrolled in the registry. In 12 patients a genetic defect associated with pigment dilution and immunodeficiency could be identified (Table I) and assigned as follows: GS2, 6 cases; Chediak-Higashi syndrome, 4 cases; and Hermansky-Pudlak syndrome type 2, 1 case. Unexpectedly, we found biallelic *PRF1* mutations in 1 patient with albinism. The association between albinism and FHL type 2 was never reported and appears to be noncausal.^35^

We identified 7 novel mutations in the *RAB27A*, *LYST*, and *AP3B1* genes. Among these, 3 were missense mutations, and all were predicted by bioinformatics facilities as damaging protein function. In 2 cases we observed a single variation: patient UPN241 has a stop mutation in *RAB27A*, with protein study showing a protein defect, and patient UPN860 has a single mutation in *LYST*, an intronic defect that is predicted by the software Human Splicing Finder to create a new acceptor site. Full characterization of these patients has yet to be completed.

### Patients with FHL with partial albinism with unassigned genetic markers

For 9 patients, a genetic marker in one of the pigment dilution–associated genes (or one of the FHL-related genes) could not be assigned (Table I). In 2 siblings (patients UPN42 and UPN43) the genetic study (as well as the functional studies) could not be performed because of lack of consent. Two patients had findings suggestive of an underlying genetic defect (ie, defective degranulation at GRA [patient UPN540] or defective cellular cytotoxicity [patient UPN244]). Another patient with no assigned marker (patient UPN299) had HLH at 2.5 years of age (with normal GRA and cytotoxicity but abnormal T-cell proliferation after CD3 stimulation), which resolved after initial treatment. This patient was later given a diagnosis of a familial depigmentation syndrome combined with recurrent infections. The family of patient UPN299 is currently under investigation for identification of a possible novel defect. The remaining 4 patients had either normal degranulation (n = 2) or normal cytotoxicity (n = 1) or were not investigated. The unassigned patients will be subject to exome sequencing in the near future.

### Analysis of pigmentation dilution in patients with FHL with partial albinism

Microscopic analysis of hair for pigment dilution produced varied results among subjects (Table I). All pigment granules were roughly oval, with the major axis aligned to the hair length. In patient UPN396 there were fine pigment granules (up to about 1.5 × 0.8 μm in diameter), as in normal blond hair. In patient UPN313 there were fine pigment granules accompanied by some medium-sized granules (about 5 × 3 μm in diameter). In 2 patients (patients UPN775 and UPN907) there were large granules (about 10 × 3 to 10 × 6 μm in diameter) unevenly distributed along the hair. One of these patients (patient UPN775) also had some hairs with fine pigment granules and no large granules.

In 3 subjects (patients UPN299, UPN797, and UPN886) there were medium-sized pigment granules. In 2 of these subjects (patients UPN797 and UPN886), there were also occasional black spindle-shaped (up to about 10 × 1 or 2 μm) images close to the hair axis but not exactly axial. Given the shape and intensely black color, these images were interpreted as air-containing fissures within the hair cortex. We have not been able to define the correlation between the degree of hair depigmentation and specific *RAB27A* mutations.

### Patients with GS2 but no evidence of pigment dilution

In addition to the patients with FHL and partial albinism (defined on the basis of the partial or complete absence of normal hair color), 45 additional patients with suspected FHL (caused by either familial disease or a confirmed severe functional defect in degranulation or cytotoxicity assays) and apparently normal pigmentation were identified, in whom we did not find biallelic mutations in the FHL-related genes *PRF1*, *UNC13D*, *STX11*, and *STXBP2* (or *SH2D1A* for XLP1 and XIAP for XLP2 in male subjects). Thus we asked whether they might have mutations in *RAB27A* that could give rise to immune defects underlying HLH in the absence of pigment dilution by preserving binding to Mlph. Of them, 29 could be investigated by using mutation analysis. Analysis of the *RAB27A* gene in 6 patients from 4 unrelated families of southern European origin unexpectedly showed biallelic mutations in *RAB27A* (Table II). All of these patients carried at least 1 novel mutation. Remarkably, the p.R141_V142delinsI mutation was shared by 5 patients from 3 unrelated families with GS2 but normal hair pigmentation: 3 homozygous siblings (patients UPN154, UPN155, and UPN313), 1 patient in association with the novel missense mutation p.S163R (patient UPN324), and another patient (patient UPN226) in association with the known p.Q172Nfs mutation. Patient UPN396 carried 2 novel missense mutations (A76V and Y159C). All missense mutations were tested by using bioinformatics software (PolyPhen-2) and defined to be pathogenic. It is interesting to note that within the same family, 2 patients (patients UPN154 and 155) had a quite typical early onset of GS2, whereas the third case (patient UPN313) had the disease only after the age of 10 years. When reviewing the hair phenotype of these patients, we confirmed that none had silver-gray hair, and only 2 were reported to have some “light or blond hair.”

The results of analysis in patients UPN396 and UPN324 are shown in Fig 1, *A*, and Fig E1, which is available in this article's Online Repository at www.jacionline.org. Both exhibited a severely reduced ability to kill target cells (maximal 20% cytotoxicity) compared with a healthy donor (maximal 80% cytotoxicity). To determine whether these patients still expressed Rab27a protein, we analyzed lysates from patients' CTLs using immunoblotting. We noted that the mutations found both in patient UPN396 (A76V and Y159C) and patient UPN324 (S163R and p.R141_V142delinsI) all resulted in reduced Rab27a protein levels in lysates from patients' CTLs (Fig 1, *B*). Interestingly, the Munc13-4 protein level was unaffected (Fig 1, *B*).

### Mutations on one face of Rab27a can disrupt binding to Munc13-4 but not Mlph

The identification of missense mutations in Rab27a that affected only CTL effector function but not melanocytes offered a unique opportunity to compare the molecular function of Rab27a in cytotoxicity versus pigmentation. Because the interaction of Rab27a with Munc13-4 is required for granule secretion from CTLs and the interaction between Rab27a and Mlph is required for melanosome secretion, we hypothesized that this might be caused by mutations in Rab27a that selectively disrupted binding with Munc13-4 but not Mlph. To investigate this hypothesis, we used the structure of mouse Rab27a in complex with human synaptotagmin-like protein 2a (Slp2a) to examine how mutations A76V, Y159C, S163R, and p.R141_V142delinsI might affect potential interaction sites or the stability of the protein.^36^ The mutation A76V lies adjacent to the active site of Rab27a, where the Mg^2+^ ion binds (green sphere, Fig 2) and GTP hydrolysis occurs, suggesting that the catalytic site might be impaired by this mutation. This is consistent with previous findings that A76V is a deleterious mutation found in patients with GS2 with immunodeficiency and albinism.^37,38^ Interestingly, residues Y159, S163, and R141 all lie close to each other in the 3-dimensional structure on an outer face of Rab27a, and the structure provides insights into why mutations of these residues might disrupt a possible interaction with Munc13-4. The structure shows that Y159 forms a hydrogen bond to the carboxy oxygen of glutamate 161. When mutated to a cysteine, this bond would be lost, and the conformation of the protein would be altered. Similarly, S163 can form a hydrogen bond to the carboxy oxygen of aspartate 136, and this would be abolished by mutation to arginine (Fig 2, second inset in second row). The deletion of 3 bases in the *RAB27A* gene (c.422_424delGAG) is found in 5 of the 6 novel patients with GS2 and results in deletion of R141 and replacement of V142 by isoleucine. Interestingly, residue R141 can also form hydrogen bonds with the carboxy group of glutamate 161 (Fig 2, third inset in second row), and these bonds would no longer exist when this residue is deleted.

Although active (GTP-bound) Rab27a in CTLs and NK cells binds to the priming factor Munc13-4, in melanocytes the key effector protein of Rab27a is the synaptotagmin-like protein Mlph. Therefore we investigated the effect of these mutations on the ability of active Rab27a to bind to either Munc13-4 or Mlph to determine whether these mutations might disrupt the binding of Munc13-4 but not Mlph and explain the loss of cytotoxicity without the loss of pigmentation. We coexpressed a point mutant of Rab27a (Q78L) that lacks GTP hydrolysis activity^36,39,40^ and each of the 4 mutations (A76V, Y159C, S163R, and delR141) found in patients (Table I), together with Mlph or Munc13-4 in HEK 293 cells, and examined whether the Rab27a mutations identified affected binding to Munc13-4 and Mlph.

When Munc13-4 immunoprecipitates were probed with anti-Rab27a antibodies, neither the S163R (Fig 3, *A*, lane 4) nor the p.R141_V142delinsI (Fig 3, *A*, lane 6) mutant forms of Rab27a were able to coprecipitate with Munc13-4 as effectively as native Rab27a (Fig 3, *A*, lane 2). Immunoprecipitation with Mlph showed that Rab27a S163R also showed greatly reduced binding to Mlph (Fig 3, *B*, lane 4). However, Rab27a p.R141_V142delinsI was able to bind Mlph (Fig 3, *B*, lane 6). Therefore the combination of these alleles would result in a specific loss of Rab27a interaction with Munc13-4 but not Mlph. These results provide a possible molecular explanation for the atypical GS2 phenotype seen in patients with severe immunodeficiency but lack of a pigmentation defect in patients UPN154, UPN155, and UPN313, who were all homozygous for the mutation at R141, as well as patient UPN324, in whom the R141 mutation is found on one allele and the S163R mutation is found on the other allele. The selective loss of Munc13-4 but not Mlph binding of the p.R141_V142delinsI mutation also provides a molecular explanation for patient UPN226 because p.Q172Nfs predicts production of a truncated protein after Q172 that would likely be degraded. Because no patients' cells were available, this could not be tested.

The mutations in patient UPN396 differed, with A76V lying in the catalytic site of Rab27a and Y159C lying close to S163, which was mutated in patient UPN324. Analyzing the ability of A76V and Y159C to interact with Munc13-4 and Mlph, we found that neither A76V nor Y159C could coprecipitate Munc13-4 as effectively as active Rab27a (Fig 3, *C*), although both could coprecipitate Mlph as effectively as active Rab27a (Fig 3, *D*). These findings explain why there is a loss of cytotoxicity in UPN396 (Fig 1, *A*) without a loss of pigmentation.

## Discussion

In this study we asked whether patients with FHL with immunodeficiency but with normal pigmentation might sometimes have mutations that affected cellular cytotoxicity without affecting pigmentation. We specifically focused on mutation analysis of *RAB27A*, *LYST*, and *AP3B1* in patients with FHL with pigment dilution, as well as a cohort with no clinical evidence of pigment dilution but no mutations in the other known FHL-related genes.

The unexpected finding that 6 patients with HLH but no albinism (only “light or blond” hair in 2 patients) showed biallelic mutations in *RAB27A* supports the concept that *RAB27A* mutations should be investigated in patients with suspected FHL, even if no pigmentation defect has been reported. Notably, in all these families we found a severe immune defect, affecting degranulation and cytotoxicity.

We identified 4 mutations at A76, R141, Y159, and S163 that specifically disrupt the interaction of Rab27a with Munc13-4 but not Mlph. The mutations R141, Y159, and S163 are all close to each other in the 3-dimensional structure of Rab27a (Fig 2), and these results indicate that this face of Rab27a forms an important part of the binding site for Munc13-4. Two separate mutations reported here affect intramolecular bonds to residue 161 in Rab27a: R141 precedes helix α4 (purple), whereas residue Y159 lies just after. Therefore it is possible that both R141 and Y159, by binding to E161, affect the position of helix α4 and thus might create an interface for the interaction with Munc13-4. Interestingly, this interface is on the opposite side of Rab27a from its Slp2a-binding site, suggesting that Rab27a can bind both Slp2a and Munc13-4 simultaneously.^36^ The mutation A76V lies near the active site of Rab27a, where GTP hydrolysis occurs. The fact that this mutation disrupts Munc13-4 binding but not Mlph binding suggests that a conformational change that occurs in this area can affect Munc13-4 but not Mlph binding. Other nearby mutations (W73G) have been found to affect the GTPase activity of Rab27a while retaining Mlph binding.^19^ Although previous investigations highlighted the linear motif of Munc13-4 required for the interaction with Rab27a,^41^ the Munc13-4–binding site on Rab27a had not been defined. By examining *RAB27A* mutations that give rise to FHL with normal pigmentation, we have pinpointed a region of Rab27a that is required for interaction with Munc13-4.

Therefore our results not only demonstrate the importance of screening patients with HLH for Rab27a defects, even when pigmentation is normal, but also provide the structural basis for these distinct phenotypes by mapping the binding sites between Rab27a and Munc13-4.

**Clinical implications**

Our study highlights the need for *RAB27A* sequencing in patients with FHL without albinism, in whom a diagnosis of GS2 can be easily missed.

## Figures and Tables

**Fig E1:** Cytolytic activity of polyclonal activated NK cells from the 3 representative patients, patient UPN440 with Chediak-Higashi syndrome, patient UPN539 with GS2 with pigment dilution, and patient UPN396 with GS2 without pigment dilution, in comparison with healthy control subjects (means ± SEMs) against the 221 B-EBV target cell line.

**Fig 1:** CTLs from patients UPN396 and UPN324 show severely reduced ability to kill target cells. **A,** Percentage killing of P815 target cells by means of redirected lysis with anti-CD3 mediated by CTLs from a healthy donor (*HD*; *triangles*), patient UPN324 *(squares)*, and patient UPN396 *(circles)* after 4 hours. Each data point was run in triplicates. The image is representative of 3 independent experiments. **B,** Immunoblots of Rab27a and Munc13-4 in CTLs from a healthy donor *(HD)* and patients UPN324 and UPN396. Proteins from lysates were separated by means of SDS-PAGE, transferred onto nitrocellulose, and probed with protein-specific antibodies against Rab27a, Munc13-4, and actin. Images are representative of 3 independent experiments.

**Fig 2:** Location of amino acid mutations in patients UPN394 and UPN326. Cartoon representation of mouse Rab27a *(yellow)* in complex with human Slp2a (cyan; 3BC1^14^) viewed from the front *(left)* and turned around the y axis to the left by 90° *(middle)*. The bound GTP analog (GppNHp) is shown as an orange stick model and the magnesium ion as a green sphere, and helix 6 is highlighted in purple. *Insets* magnify the regions where mutations in patients UPN396 and UPN324 occurred, with Y159C *(top right)*, A76V *(bottom left)*, S163R *(bottom middle)*, and p.R141_V142delinsI *(bottom right)* shown.

**Fig 3:** Effect of mutations in Rab27a on binding to Mlph and Munc13-4. Immunoblots showing coimmunoprecipitations are shown. **A,** Munc13-4 with Rab27a (*lanes 1* and *2*), Rab27a-S163R (*lanes 3* and *4*), and Rab27a-R141lfs (*lanes 5* and *6*). Images are representative of 3 independent experiments. **B,** Rab27a (*lanes 1* and *2*), Rab27a-S163R (*lanes 3* and *4*), and Rab27a-R141lfs (*lanes 5* and *6*) with Mlph. Membranes were probed with specific antibodies against Rab27a *(top)* or Mlph *(bottom)*. **C** and **D,** As above but with Rab27A A76V and Y159C. Proteins were immunoprecipitated with anti-Munc13-4 or Mlph and probed for Rab27a, Munc13-4, and Mlph.

**Table I:** Main features of 21 patients with HLH and pigment dilution

Patient ID	Sex/age	Geographic origin	GRA/cytotoxicity	Mutation analysis	Hair∗	Clinical outcome
UPN169	M/7 mo	Italy	NP/reduced	*RAB27A***c.514_518delCAAGC p.Q172NfsX2;**†		13 y, cured after SCT
UPN241	F/2 mo	Italy	NP/reduced	*RAB27A* c.550C>T p.R184X second mutation not identified		12.5 y, cured after SCT
UPN539	F/12 mo	Italy	Reduced/reduced	*RAB27A***c.148_149delAGinsC p.R50Qfs**†		Died from disease
UPN731	F/11 mo	Asian	NP	*RAB27A***c.662G>A p.C221Y**†		2.8 y, alive, SCT ongoing
UPN775	M/2 mo	Italy	Reduced/NP	*RAB27A***c.514_518delCAAGC p.Q172NfsX2**∗	Gray, small and large ovoid granules	1.5 y, cured after SCT
UPN907	F/1 mo	Asian	NP	*RAB27A* c.550C>T p.R184X†	Gray, large ovoid granules	10 mo, cured after SCT
UPN440	F/24 mo	Arab	Reduced/reduced	*LYST***c.1897A>T p.K633X**†		8 y, cured after SCT
UPN698	F/16 mo	Italy	Reduced/NP	*LYST***c.2304C>G p.C768W** Second mutation not identified		Died from disease
UPN860	M/52 mo	Czech	Normal/NP	*LYST* c.6122-4C>T (splice error) Second mutation not identified		5 y, cured after SCT
UPN886	M/26 mo	Gipsy	NP	*LYST***c.8127del5ins12 p.L2709fs**†	Gray, medium granules, spindle-shaped images	Died from disease at 3 y
UPN811	M/90 mo	Australia	NP	AP3 **c.2T>G p. M1R**†		8.5 y, alive, refused SCT
UPN351	M/4 mo	United Kingdom/Afro	NP/absent	*PRF1* c.50delT p.L17Rfs c.658G>A p. G220S		11 y, cured after SCT
UPN42	M/6 mo	Italy	NP	NP		Died from disease at 10 mo
UPN43	M/3.1 y	Italy	NP	NP		Died from disease at 3.3 y
UPN379	M/not known	Italy	NP	*RAB27A WT*	Gray, small granules	Lost to follow-up
UPN244	M/6 y	Italy	NP/absent	*RAB27A WT*		18 y, cured after SCT
UPN264	F/3 mo	Italy	NP/normal	*RAB27A WT*		10.5 y, cured after SCT
UPN299	M/2.5 y	Italy	Normal/normal	*RAB27A, LYST, AP3:* WT	Gray, medium granules	12.5 y, alive, recurrent infections
UPN540	F/12 y	Italy	Reduced/normal	*RAB27A, LYST, AP3:* WT		Died from disease at 12.2 y
UPN645	M/15.5 y	United Kingdom	Normal/NP	*RAB27A, LYST, AP3:* WT		17.7 y, alive with lymphocytopenia and thrombocytopenia
UPN797	M/21 mo	Italy	Normal/NP	*RAB27A, LYST, AP3:* WT	Gray, medium granules, spindle-shaped images	Died from disease at 2 y

Novel mutations are shown in boldface. *NP*, Not performed; *SCT*, stem cell transplantation; *UPN*, Unique patient number (UPN 42 and 43 are siblings); *WT*, wild-type.

∗ Hair study: small granules = about 0.5-1.5 × 0.3-0.8 μm; medium granules = about 2-5 × 1 μm; large granules = about 10 × 3-6 μm; spindle-shaped black images = up to about 10 × 1-2 μm and were interpreted as air-containing fissures within the hair cortex rather than pigment.

† Homozygous.

**Table II:** Main features of 6 patients from 3 families with HLH but no pigment dilution in whom GS2 was diagnosed based on *RAB27A* mutations

Patient ID	Sex/age	GRA/cytotoxicity	Mutation	Hair∗	Clinical outcome
UPN154	M/6.8 mo	NP	**c.422_424delGAG p.R141_V142delinsI**†		Died from disease
UPN155	M/0.5 mo	NP/absent	**c.422_424delGAG p.R141_V142delinsI**†		Reactivated after MRD SCT; died from disease
UPN313	F/10.7 y	Reduced/reduced	**c.422_424delGAG p.R141_V142delinsI**†	Mild blond; small- and medium-sized granules	Reactivated; 16 y, cured after UD SCT
UPN324	F/4 y	Absent/absent (Fig 1)	**c.422_424delGAG p.R141_V142delinsI c.487A>C p.S163R**		Reactivated, 13 y, cured after UD SCT
UPN396	M/7.3 y	Absent/absent (Fig 1)	**c.227C>T p. A76V c.476A>G p. Y159C**	Mild blond; small-sized granules	Reactivated; 14 y, cured after UD SCT
UPN226	M/5 y	Reduced/reduced	c.514_518delCAAGC p.Q172Nfs **c.422_424delGAG p.R141_V142delinsI**		17 y, cured after SCT

Patients UPN154, UPN155, and UPN313 are siblings. Novel mutations are shown in boldface. *MRD*, Matched related donor; *NP*, not performed; *SCT*, stem cell transplantation; *UD*, unrelated donor.

∗ Hair study: small granules = about 0.5-1.5 × 0.3-0.8 μm; medium granules = about 2-5 × 1 μm; large granules = about 10 × 3-6 μm; spindle-shaped black images = up to about 10 × 1-2 μm and were interpreted as air-containing fissures within the hair cortex rather than pigment.

† Homozygous.
